RETRACTED

# Potentiated Osteoinductivity via Cotransfection with BMP-2 and VEGF Genes in Microencapsulated C2C12 Cells

**DOI:** 10.1155/2015/435253

**Published:** 2015-09-16

**Authors:** Yang Shen, Han Qiao, Qiming Fan, Shuhong Zhang, Tingting Tang

**Affiliations:** Shanghai Key Laboratory of Orthopaedic Implants, Department of Orthopedic Surgery, Shanghai Ninth People's Hospital, Shanghai Jiao Tong University School of Medicine, 639 Zhizaoju Road, Shanghai 20011, China

## Abstract

Microcapsules with entrapped cells hold great promise for repairing bone defects. Unfortunately, the osteoinductivity of microcapsules has been restricted by many factors, among which the deficiency of functional proteins is a significant priority. We potentiated the osteoinductivity of microencapsulated cells via cotransfection with BMP-2 and VEGF genes. Various tissue-derived mesenchymal stem cells and cell lines were compared for BMP-2 and VEGF cotransfection. Ethidium bromide (EB)/Calcein AM staining revealed that all of the cell categories could survive for 4 weeks after microencapsulation. An ELISA assay indicated that all microencapsulated BMP-2 or VEGF transfected cells could secrete gene products constitutively for 1 month. Particularly, the recombinant microencapsulated C2C12 cells released the most desirable level of BMP-2 and VEGF. Further experiments demonstrated that microencapsulated BMP-2 and VEGF cotransfected C2C12 cells generated both BMP-2 and VEGF for 4 weeks. Additionally, the cotransfection of BMP-2 and VEGF in microencapsulated C2C12 cells showed a stronger osteogenic induction against BMSCs than individual BMP-2-transfected microencapsulated C2C12 cells. These results demonstrated that the cotransfection of BMP-2 and VEGF into microencapsulated C2C12 cells is of potent utility for the potentiation of bone regeneration, which would provide a promising clinical strategy for cellular therapy in bone defects.

## 1. Introduction

One major obstacle encountered by clinical orthopedic practice is the repair of bone defects caused by trauma, malignant disease, and prosthetic replacement [1]. The most common approaches to repair bone defects, such as the transplantation of autologous and allogeneic bone grafts or substitution of artificial bone, exhibit many disadvantages. These disadvantages include the scarcity of supply resources, the risk of disease dissemination, and deficient osteogenesis, which lead to the delayed union or the nonunion of the bone [2–4]. However, cell microencapsulation represents a novel and promising tissue engineering strategy that involves the carrying of viable cells with biologically active molecules or genes that promote bone regeneration [5, 6].

RETRACTED

The microencapsulation technique involves the formation of a semipermeable membrane that is able to both entrap functional and feasible cells and permit the flow of nutrients inwards and the waste of interior cells outwards [7]. Historically, microencapsulation approaches were applied to many medical conditions, such as anemia, delayed growth, and diabetes [8–10]. Furthermore, because it is an immune-tolerated biocompatible therapeutic vector, microencapsulation should assist the inner cell in avoiding host immune exterminations [11]. The alginate-poly-L-lysine-alginate (APA) microcapsules first reported by Lim and Sun [12] appear to exert an immune-protective effect on entrapped cells and form a spherical shape with a smooth surface and consistent uniformity. These were considered to be suitable standards for the use of microencapsulation in cell treatment research.

Bone morphogenetic protein-2 (BMP-2), which functions as a member of the transforming growth factor-*β* superfamily, plays a vital role during osteogenic and endochondral regeneration [13–16]. Moreover, angiogenesis appears to be a prerequisite for bone rehabilitation, and vascular endothelial growth factor (VEGF) has been proposed as the most potent induction stimulus [17]. Additionally, VEGF is capable of enhancing osteoblast differentiation by interacting with BMP-2 in a series of sequential processes [18, 19]. BMP-2 is able to enhance angiogenesis by stimulating an increased expression of VEGF on osteoblast-like cells. In turn, the accelerated establishment of new blood vessels promotes the differentiation of osteoblast cells and potentiates BMP-2-mediated bone formation [20].

Therefore, we intend to determine whether the enhanced osteoinductivity created via the cotransfection of BMP-2 and VEGF can be realized in a certain type of microencapsulated cells to provide an enhanced instrument for future cellular therapeutic progress.

Furthermore, due to the limitations of the quantity or quality of entrapped engineered cells, it is critical to identify the most satisfactory transfected cell type from among the remaining unsatisfactory cell categories to achieve the highest level of secreted functional molecules. Herein, we investigated the viability of microcapsules in various tissue-derived mesenchymal stem cells, including rat bone marrow mesenchymal stem cells (BMSCs), adipose-derived stem cells (ADSCs), synovium-derived mesenchymal stem cells (SMSCs), and divergent mouse cell lines (mouse fibroblast cell line C3H10T1/2, mouse myoblast cell line C2C12, and mouse preosteoblast cell line NIH/3T3). This investigation would significantly contribute to the development of a superior platform for microencapsulated cell delivery systems.

RETRACTED

## 2. Methods and Materials

### 2.1. Cell Preparations

#### 2.1.1. Cell Culture of Rat Bone Marrow-Derived Mesenchymal Stem Cells (BMSCs)

Male Sprague-Dawley rats weighing 300 g were purchased from the Shanghai Laboratory Animal Center, Chinese Academy of Sciences. After cervical dislocation and 75% ethanol submergence for 10 min, the rats' bilateral femurs were dissected and soft tissues were removed under aseptic conditions. Metaphyses from both proximal and distant ends were removed via diaphysis into dishes at 37°C in humidified conditions with 5% CO_2_ following a flush of 10 mL *α*MEM medium (HyClone, Logan, UT, USA) containing 10% fetal bovine serum (FBS, HyClone, Logan, UT, USA), penicillin 100 U/mL, and streptomycin 100 *μ*g/mL (Gibco, Invitrogen Ltd., Carlsbad, CA, USA). Single cell suspension was created via a syringe. The culture mediums were changed every other day until the appearance of adherent BMSCs.

#### 2.1.2. Cell Culture of Rat Adipose-Derived Stem Cells (ADSCs)

Male Sprague-Dawley rats weighing 300 g were purchased from the Shanghai Laboratory Animal Center, Chinese Academy of Sciences. After cervical dislocation and 75% ethanol submergence for 10 min, rat abdominal adipose tissues were excised. After removal of red blood cells (RBC) via a phosphate-buffer saline (PBS) wash, adipose tissue was mixed with a 3x volume of 0.1% type I collagenase (Gibco, Invitrogen Ltd., Carlsbad, CA, USA) and incubated at 37°C for 50 min. Subsequently, an equal volume of complete *α*MEM culture medium was added and centrifuged. After removal of the supernatant together with the undigested adipose tissue, cell pellets were resuspended in a 5 mL complete *α*MEM culture medium and a red blood cell lysis buffer, respectively, following several filtrations through a nylon mesh screen. Single cell suspension was created via a syringe. ADSCs were cultured at 37°C in humidified conditions with 5% CO_2_, and the culture medium was changed every other day.

#### 2.1.3. Cell Culture of Rat Knee Synovium-Derived Mesenchymal Stem Cells (SMSCs)

Male Sprague-Dawley rats weighing 300 g were purchased from the Shanghai Laboratory Animal Center, Chinese Academy of Sciences. After cervical dislocation and 75% ethanol submergence for 10 min, knee synovial membrane tissues were harvested under low temperature and washed vigorously several times in a PBS wash. Smooth and shiny synovial tissues were exposed after the removal of adipose and connective tissues. Following several washes of PBS, the synovial tissues were divided into 1-2 mm^3^ pieces with sterile blades or scissors and mixed with 0.4% type I collagenase and incubated at 37°C for 4 hr. Cell pellets were then resuspended in PBS, centrifuged several times, and cultivated at 37°C in a humidified condition with 5% CO_2_. Single cell suspension was created via a syringe. Culture medium was changed every three days.

RETRACTED

### 2.2. Cell Culture of Mouse C3H10T1/2, C2C12, and NIH/3T3 Cell Lines

Briefly, mouse fibroblast cell line C3H10T1/2 and mouse preosteoblast cell line NIH/3T3 were incubated with *α*MEM culture medium and mouse myoblast cell line C2C12 was nurtured with DMEM (HyClone, Logan, UT, USA) culture medium. C3H10T1/2, C2C12, and NIH/3T3 cell lines were purchased from the Cell Bank of the Chinese Academy of Sciences, Shanghai. Each culture medium contained 10% fetal bovine serum, penicillin 100 U/mL, and streptomycin 100 *μ*g/mL at 37°C in humidified conditions with 5% CO_2_.

### 2.3. EB/Calcein AM Staining

Following rigorous abstersion with PBS, microcapsules with entrapped cells were incubated in 100 mg/L ethidium bromide (EB) solution (Sigma-Aldrich, St. Louis, MO, USA) as well as in 5 *μ*mol/L Calcein AM (Sigma-Aldrich, St. Louis, MO, USA) for 30 min at 37°C. The morphology was observed via fluorescence microscope.

### 2.4. Transfection of BMP-2 and/or VEGF Genes

The recombinant adenovirus with the human BMP-2 gene (Adv-BMP-2) transfection was kindly provided by Professor Lou [14, 21]. The recombinant adenovirus with the human hVEGFl65 gene (Adv-VEGF) transfection was previously constructed in our lab [19]. Upon reaching 90% confluence, various cells were incubated in a transfection medium containing the culture medium and the recombinant adenovirus at the required multiple of infection (MOI) (MOI = 200 for Adv-BM-2 transfection; MOI = 150 for Adv-VEGF transfection) at 37°C overnight. Infected cells were cultivated in *α*MEM culture medium supplemented with 10% FBS; the transfection medium was changed continuously.

### 2.5. Microencapsulation of Recombinant Transfected Cells

Procedures similar to those previously described were utilized [22, 23]. Briefly, after purification, a specially designed high-voltage electrostatic microcapsule generator was utilized to manufacture APA microcapsules [24]. Recombinant transfected cell pellets were resuspended in a sterile sodium alginate solution at a concentration of 3 × 10^6^/mL via a 27-gauge needle with a syringe pump. Cell suspensions were extruded as droplets and then mixed with a 1.1% Cacl_2_ solution. The exterior layer of the microencapsulated spheres was cross-linked with poly-L-lysine (PLL) (Sigma-Aldrich, St. Louis, MO, USA) for 10 min following a soak in sodium citrate for 6 min to dissolve the unpolymerized alginate used for producing microencapsulated cells. The entire procedure was carried out at 4°C. All resultant microcapsules were stored in culturing dishes under 37°C for further research.

RETRACTED

### 2.6. Measurement of Cytokine Expressions

An identical number of entrapped cells (2.5 × 10^6^/group) in microcapsules with specific transfection were seeded and incubated for 48 hr. Then, the supernatants were collected and the concentrations of BMP-2 and VEGF were measured via enzyme-linked immunosorbent assay (ELISA) kits (BioSource, Camarillo, CA, USA) according to the manufacturer's guidelines.

### 2.7. Establishment of Coculture System between Microencapsulated Recombinant Cells with BMSCs

Six-well plates were used to investigate the interplay between upper microcapsules and lower undifferentiated bone marrow mesenchymal stem cells (BMSCs) (5.0 × 10^5^ cells/well). The basement membrane of the cell culture insert (BD Falcon, NJ, USA) was an 8 *μ*m porous PET membrane, and 2 mL DMEM culturing medium was added into each well to allow the intimate communication of cytokines between the upper and lower chambers but inhibit cell penetration.

### 2.8. Alkaline Phosphatase (ALP) Activity Assay and ALP Staining

After 3 and 7 days of coculture with recombinant microcapsules and BMSCs, the lower chamber basements were first washed twice with PBS. The ALP activity was measured in differentiated BMSCs that were lysed with 1% Triton-100 through four standard freeze and thaw cycles. Next, a 50 *μ*L sample was mixed with 50 *μ*L of* p*-nitrophenyl phosphate (*p*NPP) (Sigma-Aldrich, St. Louis, MO, USA) that served as the substrate (1 mg/mL) in a 1 M diethanolamine buffer containing 0.5 mM MgCl_2_, pH 9.8, and was further incubated at 37°C for 15 min. The reaction was stopped with the addition of 25 *μ*L of 3N NaOH for each 100 *μ*L of reaction mixture. Enzyme activity was quantified via absorbance measurements at 405 nm. The intracellular total protein expression was investigated with a BCA protein assay kit (Bicinchoninic Acid Kit, Pierce Biotechnology, Thermo Fisher Scientific, Waltham, MA, USA). ALP staining was conducted with an ALP staining kit (Renbao, Shanghai, China) on day 3 and day 7. The lower stimulated cells were fixed with 4% buffered formalin for 30 s, washed twice with cold ddH_2_O, and then stained with a staining reagent for 2 hr at 37°C according to the manufacturer's instructions. Afterwards, the plates were washed rigorously with ddH_2_O and staining images were collected under a scanner (Hewlett-Packard Scanjet 2400; Hewlett-Packard, Palo Alto, CA, USA).

### 2.9. Alizarin Red Staining (ARS)

After 21 days of coincubation with microencapsulated cells and BMSCs, the lower chamber basements were first washed twice with PBS and then fixed in 4% buffered formaldehyde for 30 min. Subsequently, the fixed cells were incubated with 40 mM Alizarin Red (Sigma-Aldrich, St. Louis, MO, USA) for 15 min, followed by a thorough wash with distilled water until the abstergent water was transparent. The final staining images were obtained with a scanner (Hewlett-Packard Scanjet 2400; Hewlett-Packard, Palo Alto, CA, USA).

RETRACTED

### 2.10. Statistical Analysis

An analysis of variance (ANOVA) and post hoc analysis were performed to assess the statistical significance of the data collected. A *P* value of less than 0.05 was indicative of a statistically significant difference. All of the data were analyzed with SPSS 13.0 software (Statistical Package for the Social Sciences, Chicago, IL, USA) and are presented as the means ± SD.

## 3. Results

### 3.1. Observations of Cultured Cells

Inverted optical microscopic observations indicated that all of the nontransfected cell types demonstrated a specific morphology (Figure 1). BMSCs exhibited a rod-like or spindle-shaped formation. After 7 days of incubation, the initial cell colony increased to merge with the other clones, bringing along the adherent spindle- and rod-shaped cells (Figure 1(a)-(A)). Regarding the ADSCs, after the first inoculation of 5–7 hr, some cells began to adhere and exhibited elongated pseudopodia, thereby contributing to a spindle-like appearance. 24 hr later, the cells completely adhered to the dishes, exhibiting a fibroblast-like cell growth with a proliferative peak at 3–5 days (Figure 1(a)-(B)). The presence of SMSCs indicated apparent adherent cells with elongated or polygonal shapes. After 72 hr of cultivation, a multitude of spindle-shaped cells with small round cells scattered inside were present. Cell colony formations were detectable at around day 5 (Figure 1(a)-(C)). Optical microscopic observations of C3H10T1/2, C2C12, and NIH/3T3 cell lines (Figure 1(b)) showed an elongated cell appearance with a rapidly proliferative bioactivity.

### 3.2. Characteristics of Microcapsules and Microencapsulated Cells

The microcapsules with or without entrapped nontransfected cells generally exhibited a smooth and spherical shape with diameters of approximately 250 *μ*m (Figure 2(a)). This uniform structure enabled the collection of results that were sufficiently reliable. Further EB/Calcein AM staining revealed that, after the microencapsulation of various cell categories, the entrapped cells were capable of surviving at least 4 weeks with no evident cell death (Figures 2(b) and 2(c)), meaning that a 4-week span of observation was able to comprehensively evaluate the transition of cytokines expressions.

RETRACTED

### 3.3. BMP-2 Productions via Microencapsulated Recombinant Cells

The productions of BMP-2 cytokines were continuously collected from the supernatants of the microcapsules.  Figure 3(a) shows the relatively low amount of BMP-2 expression in all six microencapsulated cells prior to gene transfection. After transfection of BMP-2 (Figure 3(b)), C2C12 produced a higher level than any of the other cell types from the first week to the fourth week. Also, after the peak of BMP-2 generation at week 2 in microencapsulated BMP-2-transfected C2C12 cells, a statistically significant difference from the other mesenchymal stem cells was witnessed through 4 weeks consistently.

### 3.4. VEGF Productions via Microencapsulated Recombinant Cells

The productions of VEGF cytokines were consistently harvested from the supernatants of microcapsules.  Figure 3(c) demonstrates a relatively reduced expression of VEGF prior to targeted gene transfections. After the microencapsulation of the recombinant Adv-VEGF-transfected cells, the greatest generation of VEGF was exhibited in BMSCs and ADSCs during the initial three weeks (Figure 3(d)). Additionally, C2C12 expressed the third level of VEGF expression (higher than the other three cell types).

### 3.5. BMP-2 and VEGF Productions via Microencapsulated Cotransfected C2C12 Cells

Because C2C12 cells could release the most desirable level of BMP-2 and VEGF after a single transfection, the further cotransfection of BMP-2 and VEGF at a ratio of 4 : 1 was performed in C2C12 cells.  Figure 4(a) shows a significant increase in BMP-2 release after cotransfection during the first two weeks, followed by a dramatic decline from week 2 to week 4. The generation of VEGF in cotransfected microencapsulated C2C12 cells remained stable during 4 weeks and demonstrated no significant difference from the first week. Altogether, the above data revealed that the cotransfection of BMP-2 and VEGF in microencapsulated C2C12 cells could release both BMP-2 and VEGF for 4 weeks. This method could thus be utilized for further osteoinductivity assessments.

### 3.6. Potentiated Osteoinductivity via Coculture of BMSCs with Microencapsulated BMP-2/VEGF Cotransfected Cells

The above results indicated an optimal expression of BMP-2 in recombinant C2C12 microcapsules. This method was also able to generate a satisfactory level of VEGF proteins. Therefore, the advantages of the C2C12 cell line were utilized to further investigate the osteoinductivity of BMSCs via cotransfection with BMP-2/VEGF genes. An ALP activity assay, one quantitative determination method of early osteogenic differentiation, was used to evaluate the osteoinductivity of the cocultured cells. ALP revealed that recombinant cells cotransfected with BMP-2/VEGF exhibited more significant ALP activity than those cocultured with the BMP-2-transfected microcapsules group on both day 3 and day 7 (Figure 4(b)). Additionally, the ALP activity of the BMP-2 recombinant microcapsules exhibited more significant strength than the regular culture medium-treated BMSCs group for up to 7 days. Furthermore, ALP staining results demonstrated that the cotransfected microcapsules group showed strong positive staining against BMSCs differentiation, with purple blue within the cell cytoplasm and the stronger dyeing of localized cells. In contrast, weak staining was found among the BMP-2-transfected microcapsules group with barely stained signals on days 3 and 7 in the control group, which was cocultured with undifferentiated BMSCs (Figure 4(c)). As one of the angiogenic factors, VEGF alone cannot induce the osteogenic differentiation of BMSCs cells; because of this, we did not test the efficacy of C2C12 cells transfected with VEGF alone in this study.

RETRACTED

Extracellular matrix mineralization was evaluated using Alizarin Red Staining.  Figure 4(d) shows that the staining on BMSCs cocultivated with BMP-2/VEGF-transfected microencapsulated cells displayed a multitude of red nodules after a 3-week inducement. Similar staining was observed for the BMSCs that went through BMP-2 recombinant microcapsules treatment and had a slightly weak expression. Nevertheless, few positive signals were found in BMSCs mineralization in the control microcapsules intervention. This finding was consistent with a previous study that indicated that nontransfection microcapsules explicated a negligible osteoinductivity against BMSCs after a 3-week differentiation.

## 4. Discussion

In this study, we explored the cultivation of microencapsulated BMSCs, ADSCs, SMSCs, C3H10T1/2, C2C12, and NIH/3T3 cells, revealing that the microcapsules were able to provide sufficient living conditions for the inner cells. To investigate the osteoinduced capability via the cotransfection of BMP-2 and VEGF, the C2C12 cell line was chosen for further* in vitro* coculturing with BMSCs due to its optimal expressions of both BMP-2 and VEGF. After coculture with cotransfected microencapsulated C2C12 cells, the ALP activity and ARS intensity of BMSCs were stronger than the single BMP-2-transfected group, signifying that more desirable effects were achieved via the cotransfection of BMP-2 and VEGF, which promote the expressions of osteogenic markers at both the early and the late stages.

Undoubtedly, the viable cells in microcapsules should be preserved to promote functionality. Obviously, such conditions require the formation of semipermeable membranes, which on one hand shields the invasive effects exerted on the inner sensitive and functional cells and on the other hand enables both intimate communication between the entrapped cells and the movement of exterior nutritional materials that support the stable survival of the cells entrapped in the microcapsules. With such concerns in mind, our previous study found that potentiated membrane strength and biocompatibility can be accomplished via purified sodium alginate- (PSA-) based microcapsules, indicating that the biological activity of microcapsules can be enhanced through alginate modification [25]. In this study, we also entrapped various potential osteodifferentiated cell types within APA microcapsules, showing that all of the cell categories could manage to survive within the APA microcapsules for 4 weeks.

RETRACTED

In addition, we utilized APA microcapsules with rat bone marrow-derived mesenchymal stem cells transfected with the BMP-2 gene and demonstrated both the effective immune-isolation capability of microcapsules and the valid biological response induced via the consistent and efficient release of BMP-2 from recombinant microcapsules [22]. Herein, the VEGF that served as a potent angiogenesis stimulus was utilized to enhance BMP-2-induced bone formation. Initially, BMP-2 and VEGF cytokine expressions were measured via ELISA examinations after corresponding transfection into each cell type. The 4-week duration not only demonstrated a consistent release due to the successfully microencapsulated BMP-2 and VEGF transfections but also provided us with the useful information that C2C12, which released the highest level of BMP-2 and a desirable level of VEGF, can be exploited for further cotransfection study. The C2C12 cell line acts as a premyoblast cell line [26] and could be shifted towards osteoblast differentiation from myoblast differentiation with interference of the BMP-2 protein [27–29]. Moreover, Li et al. [30] proposed that C2C12 cells were able to secrete cytokines and survive within incapacious microcapsules in the long term. Therefore, further research was carried out to compare the osteoinductivity of C2C12 cells with a single gene transfection with those with a double gene cotransfection.

VEGF, as previously reported, is capable of enhancing osteoblast differentiation with the costimulus of BMP-2 through a series of sequential processes [18, 20]. Our results showed that recombinant BMP-2 and VEGF cotransfected C2C12 cells in microcapsules could release both BMP-2 and VEGF for 4 weeks. Additionally, the ALP activity, ALP staining intensity, and ARS staining of C2C12 cells cotransfected with BMP-2 and VEGF (when examined after the 3-day and 7-day coincubation periods) demonstrated a stronger tendency than BMSCs cocultured with merely BMP-2-transfected cells, which indicated the facilitation of osteodifferentiation via the coculture of BMP-2 and VEGF cotransfected microcapsules in both the early and the late stages.

RETRACTED

Nonetheless, despite the comprehensive observation of BMSC differentiation via secreting cytokines from recombinant microcapsules, the impact on the entrapped cells after microencapsulation is not yet fully understood. SOX-9 and TGF-*β*3-transfected MSCs after microencapsulation differentiated towards cartilage, indicating that a three-dimensional culturing system of microcapsules could provide entrapped cells with an adequate microenvironment for proliferation and differentiation [31, 32]. Additionally, another study found that polysaccharide microcapsules, when used as a scaffold-based culture platform, were able to reinforce the adhesion and growth of hBMSCs [33]. Furthermore, the new bone regeneration could be unraveled after microencapsulation cultivation both* in vitro* and* in vivo* [33]. It is thus no surprise that the cellular events occurring inside microcapsules play an important role in microcapsules as an effective drug delivery vector.

In conclusion, we successfully attempted the cultivation of microencapsulated BMSCs, ADSCs, SMSCs, C3H10T1/2, C2C12, and NIH/3T3 cells with long-term lifespans. Moreover, the transfection of BMP-2 and VEGF into targeted microencapsulated cells can effectively facilitate the release of functional proteins from microcapsules. More importantly, the BMSCs' ability to differentiate can be significantly potentiated through the cotransfection of BMP-2/VEGF into C2C12 cells. This provides promising opportunities for cellular therapy in future clinical treatments of bone defects.

## Figures and Tables

**Figure 1:** The morphology of different tissue-derived mesenchymal stem cells and cell lines. (a) The morphology of different tissue-derived mesenchymal stem cells with the appearance of a colony-forming unit. (A) indicates the bone marrow-derived mesenchymal stem cells (BMSCs), (B) indicates the adipose-derived stem cells (ADSCs), and (C) indicates the synovium-derived mesenchymal stem cells (SMSCs). (b) The morphology of different cells lines. (A) represents the C3H10T1/2 cells, (B) indicates the C2C12 cells, and (C) indicates the NIH/3T3 cells. Scale: 20 *μ*m.

**Figure 2:** The morphology of APA microcapsules and the viability of various microencapsulated cells at 1 week or 4 weeks after microencapsulation (EB/Calcein AM staining). (a) The morphology of APA microcapsules. (A) indicates the microcapsules without cells and (B) indicates the microcapsules containing the BMSCs. Scale: 100 *μ*m. (b) The viability of different microencapsulated tissue-derived mesenchymal stem cells at 1 week and 4 weeks (EB/Calcein AM staining). The green fluorescence indicates live cells, and the red fluorescence indicates dead cells. Left: BMSCs, middle: ADSCs, and right: SMSCs. Scale: 20 *μ*m. (c) The viability of different microencapsulated cells lines at 1 week and 4 weeks (EB/Calcein AM staining). The green fluorescence indicates live cells, and the red fluorescence indicates dead cells. Left: C3H10T1/2, middle: C2C12, and right: NIH/3T3. Scale: 20 *μ*m.

RETRACTED

**Figure 3:** Measurement of cytokine expressions. (a) The basic BMP-2 secretion from the microencapsulated cells without gene transfection. (b) All encapsulated BMP-2 gene-transfected stem cells were capable of the constitutive secretion of BMP-2 proteins. Among the six cell types, C2C12 could secrete most BMP-2 protein, which was significantly higher than the other cell groups through four weeks after BMP-2 gene transfection and cells microencapsulation (^#^ *P* < 0.05 compared with the C2C12 group). Among the three tissue-derived MSCs, BMSCs could secrete most BMP-2 protein (significantly more than the other stem cells groups through four weeks after BMP-2 gene transfection and cells microencapsulation) (^#^ *P* < 0.05 compared with the C2C12 group). (c) The basic VEGF secretion from the microencapsulated cells without gene transfection (^#^ *P* < 0.05 compared with the C2C12 group). (d) All microencapsulated VEGF gene-transfected stem cells were capable of the constitutive secretion of VEGF proteins. BMSCs or ADSCs could secrete most VEGF proteins. C2C12 cells expressed the third level of VEGF (^#^ *P* < 0.05 compared with the C2C12 group).

**Figure 4:** Assessment of potentiated osteoinductivity. (a) Measurement of cytokine expressions after the cotransfection of BMP-2 and VEGF in microencapsulated C2C12 cells. After the cotransfection of BMP-2 and VEGF in C2C12 cells, the microencapsulated C2C12 cells could release both BMP-2 and VEGF over a span of four weeks (^#^ *P* < 0.05 compared with the 1-week observation time point). (b) The ALP activity of BMSCs cocultured with the microencapsulated C2C12 cells. BMP2 + VEGF: cocultured with the microencapsulated BMP-2 and VEGF gene-transfected C2C12 cells. BMP2: cocultured with the microencapsulated BMP-2 gene-transfected C2C12 cells. Control: coculture with the microencapsulated C2C12 lacking gene transfection (^#^ *P* < 0.05). (c) The ALP staining of BMSCs cocultured with microencapsulated C2C12 cells. (A) showed the staining results after 3 days of coculture. (B) showed the staining results after 7 days of coculture. (1) Cocultured with the microencapsulated BMP-2 and VEGF gene-transfected C2C12 cells. (2) Cocultured with the microencapsulated BMP-2 gene-transfected C2C12 cells. (3) Cocultured with the microencapsulated none gene-transfected C2C12 cells. (d) The Alizarin Red Staining of BMSCs cocultured with the microencapsulated C2C12 cells. (A) Cocultured with the microencapsulated BMP-2 and VEGF gene-transfected C2C12 cells. (B) Cocultured with the microencapsulated BMP-2 gene-transfected C2C12 cells. (C) Cocultured with the microencapsulated C2C12 cells lacking gene transfection.
